The article "Influence of HP Financial Economic Effect on Environmental Visualization under Sustainable Development" was retracted in 2023. Reasons: unreliable results or conclusions; concerns about the data; concerns about the peer review; concerns about the citations.

# Influence of HP Financial Economic Effect on Environmental Visualization under Sustainable Development

**DOI:** 10.1155/2022/7891516

**Published:** 2022-09-05

**Authors:** Jiayi Yu

**Affiliations:** School of Finance, Harbin University of Commerce, Harbin 150028, Heilongjiang, China

## Abstract

With the proposal of a sustainable development strategy, HP Finance has received extensive attention in the market, and its economic effects have also promoted the vitality of social development. However, the core of sustainable development is to achieve a two-dimensional balance between economic effects and the environment. In recent years, ecological and environmental problems have become more and more prominent and continue to bring challenges to the sustainable development of society. Environmental visualization plays an increasingly important role in the development of the times. Only by understanding the influencing factors of environmental visualization and promoting the healthy development of environmental visualization can social development goals be achieved. In the context of the social implementation of sustainable development strategies, this article deeply studies the impact of HP's financial economic effects on environmental visualization. Based on analyzing the development characteristics and status quo of the two, a fixed-effect model and a spatial model were constructed, and the specific impact of economic effects on environmental visualization was further explored. It was found through regression analysis that the breadth of coverage of economic effects and the depth of use improved the development efficiency of environmental visualization at the significance level of 0.05, respectively. However, the degree of opening to the outside world and the industrial structure in the economic effect hindered the development of environmental visualization. Its regression coefficients were −0.142, −0.134 and −0.527, −0.537. In the regression analysis of the spatial effect with a significance level of 0.01, the HP financial economic effect could promote the development of local environmental visualization, but it also hindered the development of adjacent environmental visualization. It shows that only the balanced development of economic efficiency among various regions can promote the positive improvement of the level of environmental visualization.

## 1. Introduction

The contradiction between economic development and ecological environment has always been an important issue that needs to be faced at all stages of social development. In the context of the rapid development of social modernization, ecological and environmental problems have become increasingly prominent, and environmental pollution has become increasingly serious. As a necessary means of understanding environmental information, environmental visualization can more intuitively and truly display the status quo of the ecological environment. However, environmental visualization has the characteristics of high technical requirements, high technical requirements, and high uncertainty and is a capital-intensive investment. It is difficult to meet the funding needs with its own funds or government financial support. At the same time, due to the limitations of the current social structure and other deep-seated problems (including the imperfect financial system, insufficient development of the financial market, and unbalanced supply and demand), the supply of the traditional financial sector is relatively scarce, and financing constraints have become a major obstacle to the development of environmental visualization. The emergence of HP Finance has eased the obstacles to the development of environmental visualization. In recent years, HP Finance has been vigorously developed as an important part of promoting social and economical construction. And with its advantages of low cost and high efficiency, it has promoted the stable development of a high-quality social economy. Under the sustainable development strategy, the issue of the ecological environment has always been a concern. In order to promote the in-depth development of environmental visualization, it is very important to deeply study the impact of HP's financial economic effects on environmental visualization.

The article "Influence of HP Financial Economic Effect on Environmental Visualization under Sustainable Development" was retracted in 2023. Reasons: unreliable results or conclusions; concerns about the data; concerns about the peer review; concerns about the citations.

In recent years, many scholars have deeply studied the impact of HP's financial economic effect on environmental visualization. Jin discussed the benign impact of HP's financial economic effect on poverty alleviation and environmental visualization [1]. Zheng and Xie reviewed the predicament of the rural development environment based on the background of Hewlett-Packard Finance and put forward corresponding countermeasures and suggestions [2]. Zhang et al. believed that the differences between different time dimensions in the economy and society had a certain impact on environmental visualization [3]. Chun identified and revealed the coupling relationship between urban development and ecological environment visualization under the HP financial economic effect and its formation mechanism and then proposed control measures conducive to urban management decision-making [4]. Gupta and Dutta analyzed the steady-state economic effects, which indicated that economic development could increase the level of capital stock and national income and affect environmental quality under the new steady-state equilibrium [5]. Liang used the economic index and industrial structure upgrading coefficient to study the influence of HP financial economic effect on industrial structure upgrading, such as environmental visualization [6]. The impact of HP's financial economic effect on environmental visualization covers a wide range, and previous research conclusions are relatively one-sided, unable to reveal the complex impact of HP's financial economic effect on the development of environmental visualization in the new era and the relationship between the two. From the perspective of sustainable development, it has very important times value to study it.

The article "Influence of HP Financial Economic Effect on Environmental Visualization under Sustainable Development" was retracted in 2023. Reasons: unreliable results or conclusions; concerns about the data; concerns about the peer review; concerns about the citations.

As a new mode of economic growth, sustainable development is the development requirement of the ecological environment for social economy, science, politics and many other aspects. Feris explored good governance decisions in environmental governance in the context of sustainable development and understood the way courts assess authorities' environmental decisions [7]. Franca et al. proposed a business model design method based on sustainable development strategy, which linked an organization's sustainable vision, strategy and business model [8]. Haque and Ntim observed corporate environmental performance and greenhouse gas emissions under the sustainable development framework and found that the sustainable development framework has a positive impact on environmental performance [9]. In view of the relatively limited research on multinational corporations and the SDGs, Kolk et al. discussed the important role played by multinational corporations in the SDGs [10]. Caiado et al. proposed a framework for innovative development through eco-efficiency indicators in the context of sustainable development and highlighted the coordination role between sustainable development and eco-efficiency [11]. Van de Pas explored the realities of global health governance in the context of the early implementation of the SDGs and stated that there was a governance gap between global health and development policy practices [12]. In the context of sustainable development, these studies have conducted diversified discussions on nature and the economy. However, with the continuous improvement of the economic level, environmental development also tends to be more complicated. The impact of HP financial economic effects on environmental visualization under sustainable development has important research significance.

In the context of sustainable development, this article deeply studies the impact of HP's financial economic effects on environmental visualization. Through regression analysis, it is found that at the level of significance of 0.05, the regression coefficient of HP's financial economic effect development level reaches 0.2937. The economic opening degree and the regression coefficient of the industrial structure are −0.142, −0.134 and −0.527, and −0.537, respectively, in the two dimension indexes, which hinders the healthy development of environmental visualization. There is a positive coefficient between the government and the development level of economic effects and a negative coefficient for human resources, but they are not significantly correlated. In the analysis of the spatial model, whether under the inverse distance square matrix or the economic distance matrix, the impact of the HP financial economic effect on the local environment visualization is significantly positive at the 0.01 level, and the impact on the neighboring environment visualization is significantly negative at the 0.01 level. It shows that HP's financial economic effect has a negative effect on the development of neighboring environment visualization while promoting the healthy development of local environment visualization.

The article "Influence of HP Financial Economic Effect on Environmental Visualization under Sustainable Development" was retracted in 2023. Reasons: unreliable results or conclusions; concerns about the data; concerns about the peer review; concerns about the citations.

## 2. HP Financial and Environmental Visualization

### 2.1. HP Financial Overview

The concept of HP Finance was first proposed in the China Microcredit Union in 2005 and has been mentioned many times since then. Among them, the most widely accepted related concept is a financial system for all groups and strata of society that can provide efficient services at affordable costs [13]. It is also a financial system that organically combines decentralized small financial organizations with service organizations and integrates with the entire financial development strategy. Hewlett Packard Enterprise has grown far beyond microfinance and microfinance, and its focus is that it has moved beyond a decentralized financial services organization. It aims to build an integrated financial system that integrates small and marginal microfinance systems into the formal financial system, which means there will be greater integration and more other financial institutions will join it. It not only enables different target groups to have more choices of financial products but also improves the quality of the development environment of financial services. The system is shown in Figure 1.

From the overall point of view, the HP financial situation in each province is developing well. Taking the five eastern cities as an example, the 2019–2020 HP financial index is shown in Table 1.

Judging from the growth rate of the financial index, the development of HP Finance in the market has become more and more mature in recent years. Even if it was affected by the epidemic in 2020, it still maintains positive growth, which means that HP Finance plays an important role in alleviating the economic impact of the epidemic.

The article "Influence of HP Financial Economic Effect on Environmental Visualization under Sustainable Development" was retracted in 2023. Reasons: unreliable results or conclusions; concerns about the data; concerns about the peer review; concerns about the citations.

With the rapid development of information technology in recent years, HP Finance is also catering to the development of the times in a more intelligent way, greatly reducing the cost of financial development. At the same time, information technology can not only quickly and conveniently understand the functions and usage conditions of financial services through mobile terminals and better simplify the steps and operations in the financial transaction process but also effectively integrate the information resources of service objects. It can better serve the financial industry, effectively reduce the time cost, improve the operational efficiency of financial services, and greatly increase the opportunities for social groups to obtain financial services [14].

### 2.2. Environmental Visualization Development

The original way of visualizing the environment was a simple map drawn from a piece of paper. Buildings of great reference value and significance are marked on the map, and roads are delineated according to the set ratio, which is convenient for land management in various regions and internal and external transactions. This is the earliest human cognition of the concept of environmental visualization, as shown in Figure 2.

In the future, with the opening of the economy, the exchanges between countries in the world have become more and more frequent, and the changes in the environment have become more and more complicated. Maps have become no longer simple, and more and more environmental information and data are recorded, including population density, military distribution, climate change and more. As shown in Figure 3, in addition to this one-dimensional information, some two-dimensional environmental information is also collected, analyzed and summarized on the map. For example, human beings record solar terms and observe the climate conditions in different seasons and places of the year so as to give certain guidance to social production and life. The accumulation of environmental data in different periods and different regions strengthens the accumulation of environmental data in time and space.

Due to the increasing amount of environmental information, the dimension has been extended from the traditional one-dimensional basis to two-dimensional and three-dimensional. The complexity is getting higher and higher, and a single flat map can no longer meet the development needs of environmental visualization [15]. Today, with the gradual maturity of science and technology, data processing and data simulation technology have played their own unique application value in many professional fields. Environmental researchers also use appropriate techniques to model, process, and summarize environmental information. During this period, the monitoring and simulation process of environmental data is often presented quantitatively by complex and intuitive scientific graphics, which can only be understood by relevant professionals. The process of drawing is extensive, and it pays attention to details. Once it is made, it cannot be reused, and the technical cost is also huge, which requires a huge cost. With the excavation of a large number of science and technology (Matlab and other technologies), the cost of making scientific maps has been alleviated to a certain extent. There are more and more types of maps, and more and more information can be provided, which can meet the needs of scientific researchers to a certain extent.

The article "Influence of HP Financial Economic Effect on Environmental Visualization under Sustainable Development" was retracted in 2023. Reasons: unreliable results or conclusions; concerns about the data; concerns about the peer review; concerns about the citations.

With the development of environmental science, under the background of sustainable development, it is more and more urgent to transmit environmental information to the public, popularize the status quo of environmental science development, promote the formulation and implementation of environmental protection policies, and the public's need for the effectiveness of environmental monitoring. The masses hope to feel the changes in environmental information and the meanings they represent in a more scientific and intuitive way. Therefore, it is hoped to achieve this by studying the impact of HP financial economic effects on environmental visualization. Through impact research, the development of environmental visualization is analyzed from a more in-depth perspective, which provides more scientific and reliable decision-making and a basis for its development.

### 2.3. Impact of HP Financial Economic Effects on Environmental Visualization

The characteristics of high technology content and high investment in environmental visualization determine the lack of financial support and free funds for enterprises. HP Finance has the advantages of wide coverage, low cost, and low threshold, which well meet the development needs of environmental visualization, as shown in Figure 4. On the one hand, the inclusiveness of HP Finance has eased the financing constraints of technology companies, especially for small- and medium-sized technology companies. On the other hand, relying on information technology, such as big data, cloud computing, and artificial intelligence, HP Finance has unparalleled advantages in data processing and analysis and has been applied in the fields of risk rating, investment matching, dynamic pricing, and intelligent decision-making. It has realized the role of preventing technological innovation risks and improving innovation capital security. HP Finance can communicate the supply side and the consumer side [16]. By connecting the production port and the consumer terminal of the product, the consumer's product demand can be directly fed back to the producer, which promotes the flow of information, forces enterprises to innovate, and improves the pertinence of innovation. At the same time, with the help of the networked sales platform, the digitization of production factors has been further deepened, and the logistics, capital flow, and information flow have been further integrated so as to improve the efficiency of environmental visualization products in the market. Therefore, HP Finance can stimulate the development vitality of environmental visualization and improve development efficiency. The research hypothesis of this article is that under the background of sustainable development, the development of the economic effect of HP Finance can promote the improvement of environmental visualization.

The article "Influence of HP Financial Economic Effect on Environmental Visualization under Sustainable Development" was retracted in 2023. Reasons: unreliable results or conclusions; concerns about the data; concerns about the peer review; concerns about the citations.

By constructing the fixed-effect model and spatial model of the HP financial economic effect total index on the development of environmental visualization, the impact analysis is carried out. The fixed-effect model is expressed as follows [17]:

(1) $$\begin{array}{c} evd_{it}=\beta_{1}dl_{it}+\gamma_{1}{\text{control}}_{it}+v_{i}+\varphi_{t}+\mu_{it},\\ evd_{it}=\beta_{2}bc_{it}+\gamma_{2}{\text{control}}_{it}+v_{i}+\varphi_{t}+\mu_{it},\\ evd_{it}=\beta_{2}ud_{it}+\gamma_{3}{\text{control}}_{it}+v_{i}+\varphi_{t}+\mu_{it}. \end{array}$$

Among them, *evd*_*it*_ is the development of environmental visualization and d*l*_*it*_ is the development degree of HP's financial economic effect. At the same time, on the basis of the total index, this article further considers the influence of the two dimension indexes of HP financial economic effect coverage breadth index *bc*_*it*_ and uses the depth index *ud*_*it*_ on the development of environmental visualization. *v*_*i*_ is the individual effect, *φ*_*t*_ is the time effect, *μ*_*it*_ is the error term, and control_*it*_ is the control variable, as shown in Table 2.

The spatial econometric model analyzes the spatial impact of HP financial economic effects on environmental visualization. To explore the impact of HP Finance on the development of local environment visualization and neighboring environment visualization, its model is expressed as follows [18]:

(2) $$\begin{array}{c} evd_{it}=\partial_{1}+\rho_{1}\overset{N}{\underset{j=1}{\sum }}w_{ij}evd_{it}+\beta_{1}dl_{it}+\alpha_{1}{\text{control}}_{it}+\lambda_{1}\overset{N}{\underset{j=1}{\sum }}w_{ij}x_{ij}+v_{i}+\varphi_{i}+\varepsilon_{it},\\ evd_{it}=\partial_{2}+\rho_{2}\overset{N}{\underset{j=1}{\sum }}w_{ij}evd_{it}+\beta_{2}bc_{it}+\alpha_{2}{\text{control}}_{it}+\lambda_{2}\overset{N}{\underset{j=1}{\sum }}w_{ij}x_{ij}+v_{i}+\varphi_{i}+\varepsilon_{it},\\ evd_{it}=\partial_{3}+\rho_{3}\overset{N}{\underset{j=1}{\sum }}w_{ij}evd_{it}+\beta_{3}ud_{it}+\alpha_{3}{\text{control}}_{it}+\lambda_{3}\overset{N}{\underset{j=1}{\sum }}w_{ij}x_{ij}+v_{i}+\varphi_{i}+\varepsilon_{it}. \end{array}$$

Among them, *evd*_*it*_ still represents the development of environmental visualization; *∂* is the intercept term; *ρ* is the spatial correlation coefficient, indicating the spatial correlation of the explained variables in different regions; ∑_*j*=1_^*N*^*w*_*ij*_*evd*_*it*_ is the spatial lag term; *w*_*ij*_ is the spatial weight matrix; *β* is the coefficient of the explanatory variable; d*l*_*it*_ is the total HP financial index; *bc*_*it*_ is the coverage of economic effects; *ud*_*it*_ is the depth of use of economic effects; *λ* is the spatial effect coefficient, which represents the spatial correlation of explanatory variables in different regions. ∑_*j*=1_^*N*^*w*_*ij*_*x*_*ij*_ is the spatial lag term, *v*_*i*_ is the individual effect, *φ*_*i*_ is the time effect, and *ε*_*it*_ is the random disturbance term.

The article "Influence of HP Financial Economic Effect on Environmental Visualization under Sustainable Development" was retracted in 2023. Reasons: unreliable results or conclusions; concerns about the data; concerns about the peer review; concerns about the citations.

In order to ensure the robustness of the results, in terms of the spatial weight matrix *w*_*ij*_, the geographic inverse distance square matrix *m*_1_ and the economic distance matrix *m*_2_ are selected.

In the geographic inverse distance square matrix *m*_1_, the closer the distance between regions, the greater the impact of economic effects on environmental visualization, and vice versa. The formula is expressed as follows [19,20]:

(3) $$\begin{array}{c} m_{1ij}=\left\{\begin{array}{cc} \frac{1}{d^{2}}, & \left(i\neq j\right),\\ 0, & \left(i=j\right). \end{array}\right. \end{array}$$

Among them, *d* is the centroid distance between regions.

In the economic distance matrix *m*_2_, the level of economic development is measured by the capital stock in the sample period and expressed as follows [21, 22]:

(4) $$\begin{array}{c} m_{2}=m_{1}\text{diag}\left(\frac{\bar{ed_{1}}}{\bar{ed}},\frac{\bar{ed_{2}}}{\bar{ed}},\ldots \frac{\bar{ed_{n}}}{\bar{ed}}\right),\\ \bar{ed_{i}}=\frac{1}{t_{1}-t_{0}+1}\overset{t_{1}}{\underset{t=t_{0}}{\sum }}ed_{it},\bar{ed}=\frac{1}{n\left(t_{1}-t_{0}+1\right)}\overset{n}{\underset{i=1}{\sum }}\overset{t_{1}}{\underset{t=t_{0}}{\sum }}ed_{it}. \end{array}$$

Among them, $\bar{ed_{i}}$ is the average capital stock of the region over the years. The selection of other control variables is the same as that of the fixed-effect model.

The article "Influence of HP Financial Economic Effect on Environmental Visualization under Sustainable Development" was retracted in 2023. Reasons: unreliable results or conclusions; concerns about the data; concerns about the peer review; concerns about the citations.

## 3. Empirical Results

In order to deeply understand the impact of HP's financial economic effect on environmental visualization under sustainable development and to prove the research hypothesis of this article, this article uses the fixed-effects model and spatial model to study the development of HP's financial economic effect and environmental visualization in a city. Before conducting the empirical results analysis, the city's HP financial index for the past 5 years was investigated, as shown in Table 3.

As can be seen from Table 3, the development of HP Finance in this city was relatively stable, with an average annual increase of 8.02% in the financial index based on a 5-year net growth rate. The city's HP financial economic effect development has changed from a high-speed growth stage to a normal growth stage.

In order to alleviate the problem of heteroscedasticity between variables and make the model setting more reasonable in the analysis of the impact of HP financial economic effects on environmental visualization in the context of sustainable development, logarithmic processing was performed on the model variables, as shown in Table 4.

### 3.1. Fixed-Effects Model Analysis

Regression analysis of environmental visualization was performed at a significance level of 0.05 using the two dimensions of HP financial economic effect coverage and depth of use. The regression results are shown in Figure 5.

From the regression analysis results of the two dimensions in Figure 5, it can be seen that at the level of significance of 0.05, the HP financial economic effect promotes the development of environmental visualization. Through calculation, the regression coefficients at this time reached 0.2937, respectively. The breadth of coverage of economic effects and the depth of use were at the level of significance of 0.05, respectively, and the development efficiency of environmental visualization was improved. With the expansion of its coverage and the deepening of its use, it has played a positive role in the development of environmental visualization. Both the coverage dimension index and the depth dimension index were used to verify the hypothesis of this article; that is, the HP financial economic effect can promote the development of environmental visualization.

Judging from the six control variables, under sustainable development, the role of HP's financial economic effect on infrastructure has a positive impact on environmental visualization. The improvement of the infrastructure level helps the circulation of information elements and realizes the innovative development of environmental visualization technology. The economic openness and industrial structure hinder the healthy development of environmental visualization. The regression coefficients were −0.142, −0.134 and −.527, −0.537 in the two-dimensional indices, respectively. The opening to the outside world and the improvement of the industrial structure increase the market competition for environmental visualization. Moreover, the pressure on the ecological environment has also increased significantly, which is not conducive to the healthy development of environmental visualization. The other three variables have positive and negative coefficients in the dimension index of the fixed-effects model, but they all show insignificant correlations. It shows that government expenditure, human resources, and economic development level in HP's financial economic effect have little influence on the development of environmental visualization.

The article "Influence of HP Financial Economic Effect on Environmental Visualization under Sustainable Development" was retracted in 2023. Reasons: unreliable results or conclusions; concerns about the data; concerns about the peer review; concerns about the citations.

### 3.2. Spatial Model Analysis

The use of spatial econometric models first needs to test whether the main variables have spatial correlation, and the existing research mostly uses Moran's index to test. This article uses Stata software to calculate the Moran index of HP financial economic effects and environmental visualization in 2017–2021. The results are shown in Figure 6:

It can be seen from Figure 6 that under the inverse distance square matrix, the HP financial economic effect has passed the test with a significance level of 0.05 in the five years from 2017 to 2021. The indices were 0.139, 0.182, 0.183, 0.159, and 0.174, respectively. The Moran indices of environmental visualization were 0.181, 0.126, 0.183, 0.176, and 0.193, respectively, which also passed the test with a significance level of 0.05. Under the economic distance matrix, the correlation test results of HP's financial economic effect and environmental visualization all passed the Moran test. This shows that there is a relatively obvious positive spatial correlation between HP's financial economic effect and environmental visualization, and spatial factors can be further included. The spatial model was used to further analyze the spatial effect of HP financial economic effect on environmental visualization.

Regression analysis was performed on environmental visualization at a significance level of 0.01 using the two dimensions of HP financial economic effect coverage and depth. The regression results are shown in Figure 7.

From the regression analysis results of the spatial model in Figure 7, it can be seen that whether under the inverse distance square matrix or the economic distance matrix, the impact of the HP financial economic effect on the visualization of the local environment is significantly positive at the level of significance of 0.01. It shows that the HP financial economic effect promotes the development of local environment visualization. The influence on the visualization of the neighboring environment is significantly negative at the level of significance of 0.01, indicating that the HP financial economic effect has an inhibitory effect on the improvement of the visualization of the neighboring environment. The development of the local HP financial economic effect produces a siphon effect, which inhibits the improvement of the development level of environmental visualization in the surrounding areas. At present, the financial level is still unbalanced, and the internal differentiation is serious. At the same time, the high threshold of finance strengthens the siphon effect of financially developed areas. These areas rely on their advantages in technology and capital to attract the environmental development resources of the surrounding areas and weaken the foundation for the development of financial economic effects in surrounding areas, which is not conducive to the development of environmental visualization in surrounding areas.

The article "Influence of HP Financial Economic Effect on Environmental Visualization under Sustainable Development" was retracted in 2023. Reasons: unreliable results or conclusions; concerns about the data; concerns about the peer review; concerns about the citations.

Through further analysis, whether under the inverse distance square matrix or the economic distance matrix, the coverage breadth of HP's financial economic effect and the depth of use are consistent with the sign direction of each variable, which indicates that the spatial model has good robustness. With the deepening of sustainable development, the economic effect of HP's finance is also expanding, and the gap in funding for the development of local environmental visualization can be filled, thereby improving the efficiency of scientific and technological innovation. However, due to differences in HP's financial and economic effects, there are also differences in its development environment. In areas with developed HP financial economic effects, the cost of capital use is lower, the efficiency is higher, and it is easier to promote the development of environmental visualization. At the same time, this has a side effect on the development of environmental visualization in adjacent areas.

## 4. Conclusion

Modern society pays more and more attention to the development of environmental visualization. Combined with the financial mechanism under the background of the current sustainable development era, this article deeply studies the impact of HP's financial economic effect on environmental visualization. Regression analysis is carried out on HP financial economic effect and environmental visualization through fixed-effect model and spatial model. It is found that the HP financial economic effect can effectively improve the development level and efficiency of environmental visualization at a significance level of 0.05, and its economic effect coverage breadth and depth of use have a two-way interactive impact on environmental visualization. After taking into account the space effect, it is found that the HP financial economic effect not only promotes the healthy development of local environmental visualization but also has a negative impact on the development of adjacent environmental visualization, causing a certain impact. Therefore, it is necessary to further rationally plan the development of HP Finance, narrow the differences in economic effects between regions, establish a scientific and correct concept of environmental sustainable development, and promote the benign development of environmental visualization. Of course, there are still some imperfections in the research of this article. At present, it is difficult to obtain HP financial information data. There are some limitations and incomplete considerations in the data selection in this article. And due to the lack of current empirical research, this article lacks sufficient relevant data for reference to study the impact of HP's financial economic effect on environmental visualization. In future research work, the selection of data and information will be considered from more aspects, and an analysis model with higher applicability will be constructed to improve the research level and quality.

The article "Influence of HP Financial Economic Effect on Environmental Visualization under Sustainable Development" was retracted in 2023. Reasons: unreliable results or conclusions; concerns about the data; concerns about the peer review; concerns about the citations.

## Figures and Tables

**Figure 1:** Inclusive financial system.

**Figure 2:** Simple map legend.

**Figure 3:** Information contained in the environmental visualization.

**Figure 4:** The impact of financial inclusion economic effects on environmental visualization.

**Figure 5:** Regression analysis under the dimensional index. (a) A regression analysis under the coverage index. (b) A regression analysis using the depth index.

**Figure 6:** Spatial correlation test. (a) The spatial correlation test of HP financial economic effects. (b) The spatial correlation test of environmental visualization.

**Figure 7:** Spatial effects model regression results. (a) The analysis of spatial effects under the inverse distance square matrix. (b) The spatial effect analysis under the economic distance matrix.

**Table 1:** 2019–2020 financial inclusion index.

Classification	2019	2020
Province 1	410.28	431.93
Province 2	361.93	381.61
Province 3	387.49	406.88
Province 4	330.29	350.16
Province 5	360.51	380.13

**Table 2:** Description of control variables.

Sequence	Control variable	Expression
1	Economic openness	open
2	Industrial structure	indust
3	Infrastructure	infra
4	Government spending	gov
5	Human capital	hr
6	The level of economic development	tloed

The article "Influence of HP Financial Economic Effect on Environmental Visualization under Sustainable Development" was retracted in 2023. Reasons: unreliable results or conclusions; concerns about the data; concerns about the peer review; concerns about the citations.

**Table 3:** The city's financial inclusion index for the past five years.

Areas covered	Particular year	Index
Including payment, insurance, credit services, investment, and other fields	2017	284.03
	2018	316.88
	2019	344.11
	2020	361.46
	2021	386.24

**Table 4:** Variable logarithmic processing.

Variable	Number of samples	Mean	Standard deviation	Maximum value	Minimum value
open	300	28.3614	32.0703	1.6921	149.3057
indust	300	92.0411	6.7836	71.5529	138.1693
infra	300	1.2517	0.5211	0.3743	2.7629
gov	300	2.2691	10.7466	10.7824	63.8846
hr	300	9.7922	0.8027	7.0467	14.5582
tloed	300	10.7963	0.7412	9.6538	12.6331

## Data Availability

The data used to support the findings of this study are available from the author upon request.
